# Exosomes from glioma cells induce a tumor-like phenotype in mesenchymal stem cells by activating glycolysis

**DOI:** 10.1186/s13287-019-1149-5

**Published:** 2019-02-15

**Authors:** Zhanjun Ma, Xue Cui, Li Lu, Guohu Chen, Yang Yang, Yan Hu, Yubao Lu, Zhangqi Cao, Yan Wang, Xuexi Wang

**Affiliations:** 1 The Second Clinical Medical College, Lanzhou University, Lanzhou, 730000 Gansu China; 2 The First Clinical Medical College, Lanzhou University, Lanzhou, 730000 Gansu China; 3 School of Basic Medical Sciences, Lanzhou University, Lanzhou, 730000 Gansu China; 4 Institute of Pharmacology, School of Basic Medical Science, Lanzhou University, Lanzhou, 730000 Gansu China; 5 Key Laboratory of Preclinical Study for New Drugs of Gansu Province, Lanzhou, 730000 Gansu China; 6 School of Basic Medical Sciences of Lanzhou University, School of Medicine, 205 Tianshui Rd South, Lanzhou, 730000 Gansu China

**Keywords:** Exosomes, Glioma cells, Glycolytic pathway, Tumor-like phenotype transformation, Mesenchymal stem cells, Proteomics

## Abstract

**Background:**

Exosomes are nanoscale membrane vesicles secreted by both normal and cancer cells, and cancer cell-derived exosomes play an important role in the cross-talk between cancer cells and other cellular components in the tumor microenvironment. Mesenchymal stem cells (MSCs) have tropism for tumors and have been used as tumor-tropic vectors for tumor therapy; however, the safety of such therapeutic use of MSCs is unknown. In this study, we investigated the role of glioma cell-derived exosomes in the tumor-like phenotype transformation of human bone marrow mesenchymal stem cells (hBMSCs) and explored the underlying molecular mechanisms.

**Methods:**

The effect of exosomes from U251 glioma cells on the growth of hBMSCs was evaluated with the CCK-8 assay, KI67 staining, and a cell cycle distribution assessment. The migration and invasion of hBMSCs were evaluated with a Transwell assay. A proteomics and bioinformatics approach, together with Western blotting and reverse transcriptase-polymerase chain reaction, was used to investigate the effect of U251 cell-derived exosomes on the proteome of hBMSCs.

**Results:**

U251 cell-derived exosomes induced a tumor-like phenotype in hBMSCs by enhancing their proliferation, migration, and invasion and altering the production of proteins involved in the regulation of the cell cycle. Moreover, U251 cell-derived exosomes promoted the production of the metastasis-related proteins MMP-2 and MMP-9, glioma marker GFAP, and CSC markers (CD133 and Nestin). The ten differentially expressed proteins identified participated in several biological processes and exhibited various molecular functions, mainly related to the inactivation of glycolysis. Western blotting showed that U251 cell-derived exosomes upregulated the levels of Glut-1, HK-2, and PKM-2, leading to the induction of glucose consumption and generation of lactate and ATP. Treatment with 2-deoxy-d-glucose significantly reversed these effects of U251 cell-derived exosomes on hBMSCs.

**Conclusions:**

Our data demonstrate that glioma cell-derived exosomes activate glycolysis in hBMSCs, resulting in their tumor-like phenotype transformation. This suggests that interfering with the interaction between exosomes and hBMSCs in the tumor microenvironment has potential as a therapeutic approach for glioma.

**Graphical abstract:**

ᅟ

## Background

Glioma is the most common malignant brain tumor in adults and is highly aggressive. Stem cell therapy is a new treatment option for glioma and has been evaluated in preclinical studies [1]. This approach involves the use of mesenchymal stem cells (MSCs), which can carry therapeutic factors and exert a potent anti-tumor effect [2], to alter the behavior of cancer cells.

Carcinogenesis is a multi-step, multi-factor regulatory process. Tumors consist of two principal structures: the parenchyma, or tumor cells, and the stroma, a supportive structure containing connective tissue, blood vessels [3], and macrophages, endothelial cells, lymphocytes, fibroblasts, and other mesenchymal cells. These stroma cells secrete hormones, cytokines, chemokines, and proteases to modulate the tumor microenvironment [4]. Tumor-associated stroma is a typical feature of neoplastic tissues and play a role in tumor growth, invasion, and metastasis by interacting with cancer cells [5].

MSCs are multipotent stem cells that can differentiate into stromal cells and are an important component of the tumor microenvironment. MSCs are found mainly in the connective tissue or interstitium and have marked self-renewal potential and the ability to differentiate into adipocytes, osteoblasts, and chondrocytes [6, 7]. MSCs have low immunogenicity, immunomodulatory activity, and tropism for sites of injury and inflammation and have a potential for the treatment of various diseases, including cancer [8]. These advantages have encouraged investigations of MSCs as vehicles for the delivery of anti-cancer agents [9]. However, Yu et al. [10] demonstrated that MSCs promote the proliferation and invasion of osteosarcoma cells in vitro. In addition, MSCs can promote tumor angiogenesis and may directly differentiate into pericytes and contribute to the formation of mature vasculature, thereby promoting tumor progression [11]. Therefore, reports have indicated the importance of the interaction between MSCs and cancer cells.

Tumor cells can influence MSCs via secreted factor-mediated intercellular communication. The microenvironment of the stem cell niche is a key factor in stem cell homeostasis [12]. Changes in this microenvironment may lead the transformation of normal stem cells into malignant cancer cells. For instance, Liu et al. [13] reported that exposure to the tumor microenvironment induced a tumor-like phenotype in MSCs, an effect likely mediated by factors released by the cancer cells. Moreover, cancer-derived lysophosphatidic acid stimulated the differentiation of MSCs into myofibroblast-like cells [14]. In this regard, exosomes have a vital role in this activity. These results indicate the importance of the microenvironment on MSC behavior, although the underlying mechanisms are unclear. Whether changes in the characteristics of bone marrow mesenchymal stem cells in the glioma microenvironment are caused by exosomes also remains to be determined.

Exosomes are membrane-bound vesicles of 30–120 nm secreted by various cell types, including reticulocytes, stem cells, and dendritic cells, as well as tumor cells. Exosomes contain a large number of biologically active molecules such as functional proteins, mRNAs, miRNAs, and lncRNAs. Exosomes play an important role in intercellular communication by mediating the exchange of substances and information between cells, thereby affecting the physiological functions of cells [15, 16]. Moreover, exosomes reportedly play an important role in regulating the tumor microenvironment. Exosomes released by tumor cells contain oncogenic molecules, which are important in tumor metastasis and progression, as well as the tumor-like phenotype transformation of MSCs. Indeed, exosomes released by cancer cells can be internalized by MSCs, leading to their transformation into cancer-associated fibroblasts [17–19]. In addition, lung tumor cell-derived exosomes induce the proinflammatory activity of MSCs, which promotes tumor survival [20]. However, whether glioma exosomes regulate the tumor-like phenotype transformation of MSCs is unknown.

To evaluate the risk of human bone marrow mesenchymal stem cells (hBMSCs) undergoing tumor-like phenotype transformation when used for biological therapies in the tumor microenvironment, we cultured exosomes produced by U251 cells with BMSCs. The U251-derived exosomes promoted cell proliferation, migration, and invasion and upregulated glioma-specific protein levels. A proteomic analysis indicated that U251 cell-derived exosomes induced a tumor-like phenotype in hBMSCs by activating glycolysis. These results will facilitate the clinical use of hBMSCs to treat gliomas.

## Materials and methods

### Materials

Dulbecco’s modified Eagle’s medium (DMEM)/F12 medium, fetal bovine serum (FBS), and antibiotics were purchased from Gibco/BRL (Gaithersburg, MD, USA). All reagents used for two-dimensional electrophoresis (2-DE) were obtained from Bio-Rad Laboratories (Milan, Italy), and silver staining kits were obtained from CWBIO (Beijing, China). Glucose and lactate assay kits were purchased from Nanjing Jiancheng Bioengineering Institute (Nanjing, China). The cell cycle analysis kit, Dil red fluorescence cell linker kit, and ATP assay kit were purchased from Beyotime Biotech (Nantong, China). Primary antibodies against Tsg101, CD133, Nestin, GFAP, PKLR, ANXA2, ENO1, Glut-1, HK-2, and PKM-2 were purchased from Cell Signaling Technology (Danvers, MA, USA). Antibodies against HSP70, CD9, MMP-2, MMP-9, PCNA, C-myc, and GAPDH were obtained from Proteintech Group Inc. (Chicago, IL, USA). The anti-TAGLN antibody was sourced from Abcam (UK). All other reagents were obtained from Sigma-Aldrich, unless otherwise indicated.

### Cell culture

hBMSCs were purchased from ScienCell Research Laboratories (Carlsbad, CA, USA). Human glioma U251 cells were purchased from Cyagen Biology (Santa Clara, CA, USA). Both hBMSCs and U251 cells were cultured in DMEM/F12 medium supplemented with 10% FBS and 1% penicillin-streptomycin. hBMSCs were passaged to the fourth generation for experimentation. Cells were cultured in a humidified 37 °C incubator with a 5% CO_2_ atmosphere.

### Isolation and characterization of U251 cell-derived exosomes

U251 cells were maintained in DMEM/F12 supplemented with 10% exosome-depleted FBS (EXO-FBS-50A-1, System Bioscience, Mountain View, USA) for 48 h (80–90% confluence), and the culture medium was collected and centrifuged at 800×*g* for 5 min and 1500×*g* for 15 min to remove supernumerary cells. Next, the supernatants were filtered using a Steriflip (0.22 μm, Millex-GP; Millipore, Burlington, MA, USA), and the filtrates were concentrated in a 10-kDa ultracentrifuge tube (Amicon Ultra 15; Millipore) at 4000×*g* for 30 min. U251 cell-derived exosomes were subsequently isolated using ExoQuick-TC™ (System Bioscience, Mountain View, CA, USA) according to the manufacturer’s directions. The mixture was refrigerated overnight at 4 °C and centrifuged at 1500×*g* for 30 min, and the supernatants were aspirated. The exosome-containing pellets were suspended in phosphate-buffered saline (PBS) and used immediately or stored at − 80 °C. The protein density of exosomes was measured with a BCA protein micro-assay (CWBIO, Shanghai, China). The size of exosomes was measured using a Zetasizer Nano series-Nano-ZS (Malvern Instruments, Worcestershire, UK) according to the manufacturer’s directions. The exosome markers HSP70, Tsg101, and CD9 were detected by Western blotting, and the surface markers CD63 and CD81 were detected by flow cytometry (Accuri C6; BD Biosciences, MD, USA).

### Cellular uptake of U251 cell-derived exosomes

Exosomes were labeled using a Dil red fluorescence cell linker kit according to the manufacturer’s instructions. Purified exosomes were labeled with 1 μM Dil solution for 15 min at 37 °C and washed twice with PBS to remove excess Dil. hBMSCs (50% confluence) were incubated with the Dil-labeled exosomes for 12 h in a humidified 37 °C incubator with a 5% CO_2_ atmosphere. Next, the hBMSCs were fixed with 4% paraformaldehyde for 30 min at room temperature and washed twice with PBS, and the nuclei were counterstained with DAPI for 10 min. Cellular uptake of U251 cell-derived exosomes was visualized using a Nikon Eclipse 80i confocal fluorescence microscope.

### Cell viability assay

Cell viability was assayed using the Cell Counting Kit-8 (CCK-8). hBMSCs (8 × 10^3^/well) were incubated in 96-well plates for 24 h at 37 °C. Next, the medium was changed to 100 μL DMEM/F12 medium containing 150, 300, or 600 μg/mL U251 cell-derived exosomes. Subsequently, the plates were incubated for 24, 48, or 72 h; 100 μL of fresh medium containing 10 μL of CCK-8 solution was added per well; and the plates were incubated for 30 min. The optical density at 450 nm was measured using a microplate reader (Bio-Rad, Hercules, CA, USA).

### Cell cycle analysis

hBMSCs were cultured in 25 cm^2^ plates to 40–50% confluence; the culture medium was exchanged for fresh medium containing 0.01% FBS and incubation for 24 h, which synchronizing cells. Then, the culture medium was replaced for fresh medium containing 150, 300, or 600 μg/mL U251 cell-derived exosomes, and the plates were incubated for 48 h. Next, the cells were harvested, washed twice with PBS, and fixed in ice-cold 70% (*v*/*v*) ethanol overnight at 4 °C. Subsequently, the cells were washed with PBS, stained with 500 μL of propidium iodide (50 mg/mL) in the dark for 30 min at room temperature, and analyzed by flow cytometry (Accuri C6; BD Biosciences).

### Wound healing assay

hBMSCs were cultured in 6-well cell culture plates until 70–80% confluence, and a scratch wound was created in the cell monolayer using a 200-μL pipette tip. The cells were washed twice with PBS; conditioned medium containing 150, 300, or 600 μg/mL U251 cell-derived exosomes was added: and the plates were incubated for 48 h. Images of wound healing were captured using an inverted microscope.

### Transwell assay

Cell migration and invasion were evaluated using Matrigel-coated and noncoated 24-well Transwell chambers (24-well insert; pore size, 8 μm; Corning Costar), respectively. Briefly, hBMSCs (5 × 10^4^) were added to the upper chamber of the Transwell. The hBMSCs were treated with serum-free conditioned medium containing 150, 300, or 600 μg/mL U251 cell-derived exosomes; an equal volume of exosome-depleted serum-free medium was used as the control. Complete medium containing 10% FBS (as a chemoattractant) was added to the lower chamber of the Transwell. After incubation for 48 h, the cells in the upper chamber were removed using a cotton swab and the remaining cells were fixed in 4% paraformaldehyde. The transmigrated cells were stained with 0.1% crystal violet, rinsed twice with PBS, and enumerated using an upright light microscope (Nikon, Yokohama, Japan).

### Two-dimensional gel electrophoresis and image analysis

2-DE was performed as described previously [21–23]. Briefly, after treatment with 300 μg/mL U251 cell-derived exosomes for 48 h, hBMSCs were harvested and lysed in 250 μL of lysis buffer. Whole-cell lysates (85 μg) were added to a 17-cm immobilized pH 3–10 nonlinear gradient strip (Bio-Rad Laboratories) and rehydrated in an Ettan IPG-phor isoelectric focusing system at 20 °C and 30 V for 10 h. Sample uptake into the strip was achieved at 20 °C using the following settings: 250 V for 30 min, 1000 V for 1 h, and 500 V for 10 h. Next, the strips were incubated in equilibration buffer (1% [*w*/*v*] dithiothreitol and 2.5% [*w*/*v*] iodoacetamide in 6 M urea, 0.375 M Tris-HCl [pH 8.8], 20% glycerol, and 2% sodium dodecyl sulfate [SDS]). Second-dimension separation was performed with 12% SDS-polyacrylamide gel electrophoresis (PAGE) in two steps at 10 °C: 70 V/gel for 30 min and 300 V/gel until the bromophenol blue reached the bottom of the gel. The gels were stained using a silver staining kit, and spots were detected using a GS-800 calibrated densitometer (Bio-Rad Laboratories). The images were analyzed using PDQuest™ 2-DE (ver. 8.0.1; Bio-Rad Laboratories). Protein spots were extracted from the 2-DE gels and identified with matrix-associated laser desorption/ionization-time of flight mass spectrometry (MALDI-TOF/MS) as described previously [21–23].

### Bioinformatics analysis

#### Interaction network

The protein-protein interaction network was analyzed using the STRING database ver. 10.5 (http://string-db.org).

#### Gene Ontology analysis

We analyzed the biological process (BP), molecular function (MF), and cellular component (CC) categories of the identified proteins in Gene Ontology (GO), a stratified tree structure for the examination of the functions of genes and proteins. Next, the Database for Annotation, Visualization, and Integrated Discovery (DAVID) was used to classify over-represented GO terms, and its functional annotation clustering tool was used to cluster functionally related annotations into groups. Finally, DAVID was applied to assign the identified proteins to the Kyoto Encyclopedia of Genes and Genomes (KEGG) pathways.

#### Detection of glucose consumption and lactate and ATP generation

hBMSCs were seeded in 24-well plates with 200 μL of medium per well. After incubation for 24 h, the culture medium was exchanged for fresh medium containing 150, 300, or 600 μg/mL U251 cell-derived exosomes, and the plates were incubated for 48 h. Subsequently, the supernatants and cells were harvested, and the glucose and lactate levels in the medium were determined using glucose and lactate assay kits according to the manufacturer’s instructions. Next, the hBMSCs were lysed, and the lysates were purified by centrifugation at 15,000 rpm and 4 °C for 10 min. The ATP concentration in the supernatants was measured using an ATP assay kit and a microplate reader (Bio-Rad Laboratories).

#### Immunofluorescence and nuclear staining

hBMSCs were seeded in 6-well plates and incubated with 300 μg/mL U251 cell-derived exosomes for 48 h. The cultured cells were harvested and fixed in 4% paraformaldehyde for 10 min and washed three times with PBS. Then, the cells were permeabilized using a blocking solution (5% bovine serum albumin) for 1 h. Next, the cells were incubated with anti-KI67 and anti-GFAP primary antibodies overnight at 4 °C in a dark room and detected using a FITC-conjugated secondary antibody. The nuclei were counterstained with DAPI for 10 min, and the slides were washed three times in PBS and visualized under a fluorescence microscope (Olympus, Yokohama, Japan).

#### Western blot analysis

hBMSCs were harvested and lysed in RIPA lysis buffer (Beyotime Biotech). Subsequently, protein samples (15 μg) were separated in a 12% SDS-PAGE gel, transferred to polyvinylidene difluoride (PVDF) membranes (Millipore), and blocked in Tris-buffered saline/Tween 20 solution containing 5% nonfat dry milk for 2 h at room temperature. Next, the membranes were incubated with primary antibodies against MMP-2, MMP-9, PCNA, C-myc, CD133, Nestin, GFAP, PKLR, TAGLN, ANXA2, ENO1, Glut-1, HK-2, and PKM-2 at 4 °C overnight. Thereafter, the membranes were incubated with the corresponding secondary antibodies for 1 h. Signals were visualized by chemiluminescence (Bio-Rad), and images of the blots were analyzed using ImageJ software (NIH, Bethesda, MD, USA).

The protein concentrations in U251 cell-derived exosomes were determined using a BCA protein assay kit. Exosomal protein samples (15 μg) were subjected to 12% SDS-PAGE and transferred to PVDF membranes. The membranes were incubated with Hsp70, CD9, and Tsg101 primary antibodies and visualized using a chemiluminescence substrate and gel imaging system (ImageJ software Bethesda, MD, USA).

#### Quantitative reverse transcription quantitative polymerase chain reaction

Total RNA was isolated from hBMSCs using IAzol lysis reagent (Qiagen, Valencia, CA, USA) according to the manufacturer’s instructions. Complementary DNA (cDNA) was synthesized from 1 μg of total RNA using a cDNA reverse transcription kit (TaKaRA, Dalian, China) according to the manufacturer’s instructions, and the mRNA levels of p53, NS, GFAP, Glut-1, HK-2, PKM-2, PCNA, and C-myc were determined by RT-qPCR following a standard protocol with the LightCycler 96 System (Roche, Pleasanton, CA, USA) and detection via SYBR green (SYBR Green Supermix; TaKaRa). The results were normalized to the GAPDH mRNA level. Fold change values were analyzed using the 2^−ΔΔCt^ method. The sequences of the primers are listed in Table 1.

**Table 1:** Primer sequences for qRT-PCR

Gene	Forward primer sequence	Reverse primer sequence
P21	GGATTGGTTGGTTTGTTGGAATTT	ACAACCCTAATATACAACCACCCC
P16	AACGCACCGAATAGTTACGG	CACCAGCGTGTCCCAGGAAG
MMP-2	TATGGCTTCTGCCCTGAGAC	CACACCACATCTTTCCGTCA
MMP-9	AGTCCACCCTTGTGCTCTTC	ACTCTCCACGCATCTCTGC
GFAP	GATCAACTCACCGCCAACAG	AGGTTGTTCTCG GCTTCC AG
CD133	ACAATTCACCAGCAACGAGTCC	GACGCTTTGGTATAGAGTGCTCA
Nestin	GGG AGTCCGATGGGTTTG	GGC TCCCAACAGAAGACC
Glut-1	CTTTGTGGCCTTCTTTGAAGT	CCACACAGTTGCTCCACAT
PKM-2	GGGTTCGGAGGTTTGATG	ACGGCGGTGGCTTCTGT
HK-2	TGCCAAGCGTCTCCATAA	GGTCAGCCAGACGGTAA
GAPDH	GCACCGTCAAGGCTGAGAAC	ATGGTGGTGAAGACGCCAGT

#### 2-Deoxy-d-glucose treatment

hBMSCs were treated with 300 μg/mL U251 cell-derived exosomes and 2.5 mM 2-deoxy-d-glucose (2-DG) for 48 h. To assess the proliferation, migration, invasion, and tumor-associated proteins of hBMSCs, the specific steps are the same as the above methods.

#### Statistical analysis

The data are presented as the means ± standard deviation (SD) of triplicate experiments, and the statistical significance of differences was analyzed with Student’s *t* test using SPSS ver. 21.0 software (IBM, Armonk, NY, USA). A *P* value < 0.05 was considered to indicate statistical significance.

## Results

### Characterization of U251 cell-derived exosomes

To determine whether U251 cell-derived exosomes were successfully purified, firstly, the proteins acquired from U251 cell-derived exosomes were separated by 10% SDS-PAGE and stained with Coomassie Blue. The results indicated that isolated exosomes contained a large number of proteins, which had an unlike profile (Fig. 1a). The exosomes were 20–200 nm in diameter (Fig. 1b). Western blot analysis showed that the U251 cell-derived exosomes had higher levels of HSP70, Tsg101, and CD9 than U251 cells (Fig. 1c). Using flow cytometry, we found that the exosomes were positive for CD63 and CD81 (Fig. 1d, e). Therefore, the vesicles isolated from the U251 cell culture supernatant were exosomes.

**Fig. 1:** Characterization of exosomes that originated from U251 cells. **a** The different amount (5, 10, 20, 30, and 40 μg) of protein from U251 cell-derived exosomes were loaded and run on a 10% SDS gel and stained with Coomassie Blue. **b** The size of U251 cell-derived exosomes detected by Zetasizer Nano ZS. **c** Western blot analyses of exosomal markers (HSP70, Tsg101, and CD9). **d**, **e** Flow cytometry analyses of exosomal surface markers (CD63 and CD81)

### Exosomes promote hBMSC proliferation

After incubation with fluorescent-labeled exosomes for 12 h, over 85% of the hBMSCs exhibited red fluorescence (Fig. 2a), indicating that the hBMSCs took up the U251 cell-derived exosomes. Moreover, the CCK-8 assay showed that the exosomes increased the proliferation of hBMSCs in a time- and concentration-dependent manner (Fig. 2b). In addition, Ki67 immunofluorescence staining demonstrated that exosomes significantly increased the proliferation of hBMSCs (Fig. 2c). Treatment with U251 cell-derived exosomes induced the production of PCNA and C-myc in hBMSCs (Fig. 2d, e). Flow cytometric analysis indicated that the proportion of exosome-treated hBMSCs in the S phase was greater than that of untreated hBMSCs (Fig. 2f, g). Using real-time PCR, treatment of hBMSCs with U251 cell-derived exosomes significantly downregulated p16 and p21 mRNA levels compared to the controls (Fig. 2h). Therefore, the U251 cell-derived exosomes accelerated DNA replication and promoted the proliferation of hBMSCs.

**Fig. 2:** U251 cell-exosomes promote the proliferation of hBMSCs. **a** Cellular internalization of Dil-labeled U251 cell-derived exosomes into hBMSCs. **b** hBMSCs were treated with different concentrations of U251 cell-derived exosomes for different time points (24, 48, and 72 h), and then cell viability was measured using the CCK-8 analyses. The results showed U251 cell-derived exosomes could promote hBMSC proliferation in a time- and dose-dependent manner with respect to control cells (*P < 0.05). **c** Representative images of Ki67 immunostaining in hBMSCs treated with or without U251 cell-derived exosomes for 48 h. Green fluorescence indicated the Ki67-positive cells. **d** Protein expression of PCNA and C-myc was determined by Western blotting analysis in hBMSCs treated U251 cell-derived exosomes for 48 h. **e** Bar graphs showing the relative protein expression level of PCNA and C-myc in hBMSCs treated with U251 cell-derived exosomes for 48 h. The protein levels of GAPDH served as loading controls (*P < 0.05). **f** The hBMSCs exposed with exosomes for 48 h showed an increase in the S phase of the cell cycle compared to the controls. **g** Treatment of exosomes caused a S cell cycle arrest in a dose-dependent manner, the arresting rate increased more rapid in hBMSCs exposed with exosomes than control cells for 48 h (*P < 0.05, **P < 0.01). **h** Real-time PCR analysis of P21 and P16 mRNA expression in hBMSCs treated with U251 cell-derived exosomes for 48 h (*P < 0.05, **P < 0.01)

### U251 cell derived-exosomes promote the invasion and migration of hBMSCs

The wound healing assay showed that treatment with U251 cell-derived exosomes significantly increased the wound closure rate of hBMSCs in a dose-dependent manner (Fig. 3a, b). Furthermore, the Transwell chamber assay showed that U251 cell-derived exosomes significantly increased the number of migrated and invaded hBMSCs compared to the control (Fig. 3c, d). Therefore, the U251 cell-derived exosomes increased the migration and invasion of hBMSCs in a dose-dependent manner.

**Fig. 3:** U251 cell-derived exosomes contribute to the promotion of the migration and invasion of hBMSCs. **a** The movement of hBMSCs was observed by wound healing assay at 0 h and 48 h after exosomes treatment. **b** The wound closure rate of hBMSCs was quantified by measuring wound closure areas at 0 h and 48 h (*P < 0.05, **P < 0.01). **c** The migration and invasion abilities of hBMSCs were examined by Transwell assay after treatment with U251 cell-derived exosomes for 48 h. The photos represented cell invasion into the underside of the Transwell membrane under a microscope at × 200 magnification field. **d** The hBMSC number that crossed the Transwell chamber of each group was counted and averaged after treatment with U251 cell-derived exosomes for 48 h (*P < 0.05, **P < 0.01). **e** hBMSCs were treated with 300 μg/mL U251 cell-derived exosomes for 48 h. MMP-2 and MMP-9 proteins in hBMSCs were detected by Western blotting. The ratios of MMP-2 and MMP-9 were relative to GAPDH and standardized to the control group (*P < 0.05). **f** The mRNA expression levels of MMP-2 and MMP-9 in hBMSCs treated with U251 cell-derived exosomes for 48 h (*P < 0.05)

Next, we evaluated the molecular mechanisms underlying the effect on hBMSC migration and invasion of U251 cell-derived exosomes by Western blotting and real-time RT-PCR. Exosome application increased MMP-2 and MMP-9 protein and mRNA levels (Fig. 3e–g). Therefore, the U251 cell-derived exosomes promoted the migration and invasion of hBMSCs by increasing the levels of MMP-2 and MMP-9.

### U251 cell-derived exosomes upregulate the protein levels of cancer markers

CD133 and Nestin are markers of neural stem cells and cancer stem cells (CSCs), and GFAP is a marker of glioma cells. Via immunostaining, we found that treatment with the exosomes induced GFAP expression in hBMSCs (Fig. 4a). Western blot and RT-PCR analyses showed that treatment of hBMSCs with U251 cell-derived exosomes for 48 h upregulated the protein and mRNA levels of GFAP, CD133, and Nestin in a dose-dependent manner (Fig. 4b–d). Therefore, the glioma microenvironment promotes the expression of GFAP, CD133, and Nestin, which may contribute to the tumor-like phenotype transformation of hBMSCs.

**Fig. 4:** Tumor-associated factors were induced or increased in hBMSCs by treatment with exosomes from U251 cells for 48 h. **a** Fluorescence images showing that the hBMSCs express the glioma-related marker GFAP after treatment with 300 μg/mL U251 cell-derived exosomes (× 200). **b** The protein levels of GFAP, CD133, and Nestin were examined by Western blotting after treatment with 150, 300, and 600 μg/mL U251 cell-derived exosomes. **c** Bar graphs showing the relative protein expression level of GFAP, CD133, and Nestin. The protein levels of GAPDH served as loading controls (*P < 0.05,**P < 0.01). **d** The mRNA expressions of GFAP, CD133, and Nestin. GAPDH was used as the endogenous control (*P < 0.05)

### Proteomics analysis

Next, we performed a proteomics analysis of hBMSCs treated with 300 μg/mL U251 cell-derived exosomes for 48 h. The resolution of proteins extracted from exosomes by 2D-PAGE generated reproducible pairs of 2-D gel images (Fig. 5). The ten proteins that showed at least twofold difference in intensity between the exosomes and hBMSCs (*P* < 0.05) were used for further analysis.

**Fig. 5:** 2-DE profiling of the differentially expressed proteins between hBMSCs and hBMSCs incubated with 300 μg/mL U251 cell-derived exosomes for 48 h. Total protein extracts were separated on pH 3–10 nonlinear IPG strips in the first dimension, followed by 12% SDS-PAGE in the second dimension and visualization by silver staining. **a** Representative 2-DE image of control hBMSCs for 48 h. **b** Representative 2-DE image of hBMSCs treated with 300 μg/mL U251 cell-derived exosomes for 48 h. The differentially expressed spots were identified by MS (marked with an arrow and number)

### Identification of proteins

Of the 15 protein spots, 10 were identified by MALDI-TOF/MS (Table 2). Among these 10 proteins, 6 (Annexin A2 [ANXA2], voltage-dependent anion-selective channel protein 1 [VDAC21], WD repeat-containing protein 1 [WDR1], phosphoglycerate kinase 1 [PGK1], enolase 1 [ENO1], and glucose-6-phosphate isomerase [GPI]) were upregulated and 4 (transgelin [TAGLN], pyruvate kinase [PKLR], triosephosphate isomerase [TPI1], and 14-3-3 protein zeta/delta [YWHAZ]) were downregulated. The search results for spots 1 and 5 are shown in Figs. 6 and 7.

**Table 2:** MALDI-TOF-MS/MS identification results of differentially expressed protein spots

Spot no.	Protein name	Accession no.	MW (KD)	pI	Score	Sequence coverage (%)	Matches	Expression change
1	Annexin A2	P07355	38.81	7.57	364	19	5 (5)	Increase
2	Voltage-dependent anion-selective channel protein 1	P21796	30.87	8.62	181	12	3 (3)	Increase
3	Transgelin	Q01995	23.75	8.54	323	42	9 (7)	Decrease
4	Pyruvate kinase PKLR	P30613	61.83	5.82	392	31	12 (9)	Decrease
5	Triosephosphate isomerase	P60174	26.94	6.45	179	48	10 (8)	Decrease
6	WD repeat-containing protein 1	O75083	66.82	6.17	254	52	7 (6)	Increase
7	14-3-3 protein zeta/delta	P63104	27.90	4.73	182	31	6 (4)	Decrease
8	Phosphoglycerate kinase 1	P00558	42.50	5.0	214	56	5 (3)	Increase
9	Enolase 1, (alpha)	P06733	47.59	6.44	273	21	8 (5)	Increase
10	Glucose-6-phosphate isomerase	P06744	59.13	6.40	135	44	6 (5)	Increase

**Fig. 6:** Identification of protein spot #1 from Fig. 5. **a** Output of the database searching by the MASCOT program using MS/MS data resulted in the identification of Annexin A2. **b** Protein sequence of Annexin A2 is shown. The matched peptides are in bold red. **c** Mass spectrum of tryptic peptide from spot #1

**Fig. 7:** Identification of protein spot #5 from Fig. 5. **a** Output of the database searching by the MASCOT program using MS/MS data resulted in the identification of triosephosphate isomerase. **b** Protein sequence of triosephosphate isomerase is shown. The matched peptides are in bold red. **c** Mass spectrum of tryptic peptide from spot #5

### Confirmation of the protein identification by Western blot analysis

The results of the Western blot analysis confirmed the differential levels of PKLR, TAGLN, ANXA2, and ENO1 in exosome-treated and exosome-untreated hBMSCs. Treatment with the exosomes resulted in the upregulation of ANXA2 and ENO1 protein and downregulation of PKLR and TAGLN protein in hBMSCs (Fig. 8a, b). The 2-DE and Western blot analyses yielded similar results.

**Fig. 8:** Western blot analysis to confirm the PKLR, TAGLN, ANXA2, and ENO1 in hBMSCs treated with 300 μg/mL U251 cell-derived exosomes for 48 h. **a** The PKLR, TAGLN, ANXA2, and ENO1 proteins in hBMSCs were detected by Western blotting. **b** Bar graphs showing the relative expression levels of PKLR, TAGLN, ANXA2, and ENO1 proteins. GAPDH was used as internal control (*P < 0.05)

### Bioinformatics analysis of the signaling network

Next, we used the online STRING database to predict the interaction networks among the identified proteins (Fig. 9a). ENO1, PKLR, and TPI1 were key nodes and modulators in the network. Next, the analysis of the GO function classifications of the proteins showed that 13 were annotated as MF, 97 as BP, and 23 as CC (*P* < 0.05). The top 10 significantly enriched GO terms identified by screening using a threshold false discovery rate of < 0.01 are shown in Fig. 9b–d. In addition, the proteins were enriched in the glycolysis/gluconeogenesis, carbon metabolism, biosynthesis of antibiotics, biosynthesis of amino acids, and metabolic KEGG pathways (Fig. 9e). The KEGG maps of the glycolysis/gluconeogenesis signaling pathways are shown in Fig. 9f. Therefore, the identified proteins were involved in several biological processes and showed diverse molecular functions, mainly related to the activation of the glycolysis/gluconeogenesis signaling pathway and other metabolic pathways.

**Fig. 9:** Protein interaction network and functional analysis. **a** The network containing ten identified differentially expressed proteins were mapped using the STRING system (http://string-db.org) based on evidence with different types. **b**–**d** Gene Ontology (GO) classification of the hBMSC proteins affected by U251 cell-derived exosomes. The *y*-axis shows significantly enriched Gene Ontology (GO) terms relative to the genome, and the *x*-axis shows the enrichment scores of these terms. **b** Molecular function (MF) categories in GO. **c** Biological process (BP) categories in GO. **d** Cellular component (CC) categories in GO. **e** KEGG analysis of differentially expressed proteins associated signal pathways. **f** KEGG pathway enrichment analysis maps of the glycolysis/gluconeogenesis signal pathway

### U251 cell-derived exosomes activate glycolysis in hBMSCs

Changes in cellular metabolism are important characteristics of tumors, and aerobic glycolysis promotes the survival of tumor cells [23]. Therefore, we explored the effect of U251 cell-derived exosomes on glycolysis in hBMSCs. Application of U251 cell-derived exosomes significantly increased the rate of glucose consumption, as well as those of lactate and ATP production, in hBMSCs in a dose-dependent manner (Fig. 10a–c). Moreover, the protein and mRNA levels of Glut-1, HK-2, and PKM-2 were significantly upregulated by the U251 cell-derived exosomes in a dose-dependent manner (Fig. 10d–f). Therefore, the U251 cell-derived exosomes modulated the glucose metabolism and enhanced the glycolysis in hBMSCs.

**Fig. 10:** The levels of glycolysis pathway influenced by U251 cell-derived exosomes in hBMSCs. The hBMSCs were incubated with different concentrations (150, 300, and 600 μg/mL) of U251 cell-derived exosomes for 48 h. **a**–**c** The level of glucose consumption, lactate production, and cellular ATP production were assayed. U251 cell-derived exosomes could increase the glucose consumption and lactate and ATP production compared to the control group in the hBMSCs (*P < 0.05, **P < 0.01). **d** The expression levels of several key glycolytic pathway-related proteins (Glut-1, HK-2, and PKM-2) were measured by Western blotting after hBMSCs were treated with U251 cell-derived exosomes. **e** Bar graphs showing the relative protein expression level of Glut-1, HK-2, and PKM-2. The protein levels of GAPDH served as loading controls (*P < 0.05). **f** The mRNA expressions of Glut-1, HK-2, and PKM-2. GAPDH was used as the endogenous control (*P < 0.05)

### Inhibition of glycolysis reverses tumor-like phenotype transformation of hBMSCs

To validate the finding that induction of glycolysis induces a tumor-like phenotype in hBMSCs, we used the glucose analog 2-DG, a competitive inhibitor of glycolysis. Treatment with 300 μg/mL U251 cell-derived exosomes promoted the proliferation, migration, and invasion of hBMSCs; these effects were reversed by 2-DG (Fig. 11a–c). Furthermore, Western blot analysis showed that MMP-2 and MMP-9 protein levels were decreased by 2-DG (Fig. 11d, e). Similarly, 2-DG decreased the exosome-mediated increased protein levels of PCNA, C-myc, CD133, Nestin, and GFAP (Fig. 12a–c). Therefore, inhibition of glycolysis reversed the tumor-like phenotype transformation of hBMSCs in the glioma microenvironment.

**Fig. 11:** 2-DG reversed the tumor-like phenotype transformation of hBMSCs under the treatment of U251 cell-derived exosomes. The hBMSCs were incubated with 300 μg/mL U251 cell-derived exosomes or 2.5 mmol/L 2-DG for 48 h. **a** 2-DG could suppress the proliferation of hBMSCs under the treatment of U251 cell-derived exosomes for 24 h, 48 h, and 72 h (*P < 0.05). **b**, **c** The effects of 2-DG on hBMSCs migration capability were assessed by the Transwell assay with or without Matrigel under the treatment of U251 cell-derived exosomes. The number of migrated or invaded cells was quantified by counting the number of cells from five random fields at a × 200 magnification (*P < 0.05). **d**, **e** Protein levels of MMP-2 and MMP-9 were examined by Western blotting under the treatment of U251 cell-derived exosome or 2.5 mmol/L 2-DG. GAPDH was an internal control (*P < 0.05)

**Fig. 12:** 2-DG reverses the tumor-associated factors of hBMSCs under the treatment of U251 cell-derived exosomes. The hBMSCs were incubated with 300 μg/mL U251 cell-derived exosomes or 2.5 mmol/L 2-DG for 48 h. **a** The protein levels of PCNA, C-myc, CD133, Nestin, and GFAP were examined by Western blotting. **b**–**d** Bar graphs showing the relative protein expression level of PCNA, C-myc, CD133, Nestin, and GFAP. The protein levels of GAPDH served as loading controls (*P < 0.05)

## Discussion

Solid tumors comprise tumor cells, stromal cells, inflammatory cells, vasculature, and extracellular matrix, which together form the tumor microenvironment [4]. Tumor development, metastasis, and drug resistance depend on the communication between tumor cells and their microenvironment, which can be mediated by exosomes [24]. Exosomes promote tumor formation and development by mediating the intercellular transport of oncogenes and proteins. Cancer cell-derived exosomes may exert several effects simultaneously; therefore, their biological functions are somewhat unclear [25]. In this study, we focused on the role of exosomes in the tumor microenvironment.

Paracrine and endocrine signals cause MSCs to migrate toward the sites of wounds, injury, and inflammation. MSCs can also migrate to tumors, which may be considered to be “never-healing wounds” and comprise tumor stroma [26]. Therefore, MSCs show potential as vehicles for anti-cancer agents [27]. However, exosomes produced by tumor cells are capable of influencing MSCs [28, 29]. MSCs are reportedly intimately associated with tumor cells in the tumor microenvironment; indeed, co-culture with lung cancer A549 cells promoted the proliferation and migration of hBMSCs, likely by modulating the expression of genes related to the ERK signaling pathway [30]. Furthermore, C6 glioma-conditioned medium induced a tumor-like phenotype in MSCs, possibly in a manner involving the S100B/RAGE pathway [31]. The mechanisms by which cancer cells induce MSCs to differentiate into myofibroblasts differ according to the type of cancer [32, 33]. Therefore, the interaction between MSCs and tumor cells represents a candidate therapeutic target. Although MSCs undergo tumor-like phenotype transformation in the glioma microenvironment, the underlying mechanism is unclear. Therefore, we performed a proteomics analysis to clarify the effects of U251 cell-derived exosomes on hBMSCs, as well as the underlying mechanisms.

The U251 cell-derived exosomes were efficiently taken up by, and enhanced the proliferation of, hBMSCs. Moreover, the exosomes upregulated the protein levels of PCNA and C-myc in hBMSCs. PCNA is required for DNA replication and genome maintenance in actively growing cells. Due to its role in cancer cell proliferation, PCNA is widely used as a tumor marker. Abnormal expression of PCNA is closely related to the occurrence and development of tumors and can be used to evaluate their malignant and proliferative potential [34]. C-myc is a transcriptional regulator encoded by the proto-oncogene myc; C-myc at oncogenic levels reprograms cellular metabolism, as a marker of carcinogenesis, to maintain the high rate of proliferation of cancer cells [35]. Treatment with U251 cell-derived exosomes significantly increased the proportion of S phase cells and downregulated the mRNA and protein levels of P16 and P21, negative regulators of the cell cycle in hBMSCs [36]. Therefore, the promotion by U251 cell-derived exosomes of the proliferation of hBMSCs is linked to the altered expression of C-myc and regulators of the cell cycle. Specifically, after incubation with Dil-labeled exosomes, it is found exosomes (or Dil) presented around the nucleus (or DAPI) of hBMSCs, indicating that the hBMSCs maybe take up the U251 cell-derived exosomes into the cell membrane or cytoplasm. Therefore, the specific cellular localization of exosomes-binding is still in need of further study.

We found that the U251 cell-derived exosomes promoted the migration and invasion of hBMSCs, possibly by modulating the expression of genes encoding matrix metalloproteinases (MMPs), which play an important role in tumor invasion and metastasis [37]. The U251 cell-derived exosomes also upregulated the mRNA and protein levels of MMP-2 and MMP-9 in a dose-dependent manner. We also evaluated the mRNA and protein levels of GFAP, CD133, and Nestin by immunofluorescence, Western blotting, and RT-PCR. GFAP is known to be involved in normal astrocyte functions and commonly used as a histological marker for tumors of glial origin [38]. GFAP has been previously shown to be co-expressed with nestin in glioma cells and is over-expressed in the serum and peripheral blood of glioma patients in comparison with healthy controls; GFAP staining is considered a standard diagnostic marker for glioma [38]. Moreover, nestin is expressed in several types of cancer and it is strongly associated with glioma. Increased nestin expression has been related to higher grade glioma and lower patient survival rates [39]. Meanwhile, CD133^+^ human glioma cells can initiate tumor formation in the brains of immunodeficient mice. Interestingly, these cells also express nestin, indicating the possibility of CD133 expression on progenitor cells [40]. Some reports demonstrated that nestin and CD133 are markers of neural stem cells and are used to determine the biological properties of CSCs [41]. The U251 cell-derived exosomes upregulated the mRNA and protein levels of GFAP, CD133, and Nestin in hBMSCs, suggesting that hBMSCs undergo transformation into glioma CSCs in gliomas. Accumulating evidence indicates that tumors are derived from CSCs [42], which have self-renewal potential and enhanced proliferation, thereby promoting tumorigenesis [43].

We identified the target molecules of U251 cell-derived exosomes in hBMSCs by proteomics analysis; this yielded ten proteins whose levels differed between exosome-treated and exosome-untreated hBMSCs. Among them, six proteins (ANXA2, VDAC21, WDR1, PGK1, ENO1, and GPI) were upregulated and four (TAGLN, PKLR, TPI1, and YWHAZ) were downregulated. The PKLR, TAGLN, ANXA2, and ENO1 proteomics data were verified with Western blotting.

*ENO1* encodes the enzyme responsible for the conversion of 2-phosphoglycerate into phosphoenolpyruvate and c-myc binding protein (MBP-1) [44]. Overexpression of ENO1 is related to tumor development, progression, and invasion. ENO1 promotes colorectal tumorigenesis and metastasis through the AMPK/mTOR pathway [45] and is overexpressed in lung cancer and promotes glycolysis, proliferation, metastasis, and tumorigenesis through PI3K/AKT pathway activation [46]. These reports support our finding that U251 cell-derived exosomes significantly upregulated ENO1 in hBMSCs.

ANXA2 is a membrane-bound protein expressed in most eukaryotic cells whose function is dependent on Ca^2+^ [47]. ANXA2 plays a critical role in the adhesion, migration and invasion, proliferation, and angiogenesis of tumor cells [48]. ANAX2 is reportedly overexpressed in multiple cancers and is involved in their development and metastasis [49]. Therefore, the upregulation of ANXA2 may be related to the U251 cell-derived exosome-induced tumor-like phenotype in hBMSCs.

PGK1 is the first ATP-generating enzyme in glycolysis and catalyzes the reversible transfer of 1,3-bisphosphoglycerate and ADP into 3-phosphoglycerate and ATP [50]. PGK1 is secreted extracellularly by tumor cells, and its upregulation is associated with tumorigenesis [51–53]. PGK1 regulates glycolysis, angiogenesis, and autophagy, which play vital roles in cancer metabolism and tumorigenesis [53]. In this study, treatment with U251 cell-derived exosomes upregulated PGK1 in hBMSCs, suggesting the promotion of glycolysis leading to tumor-like phenotype transformation.

Among the 10 protein spots identified, 6 were upregulated and 4 were downregulated. These proteins clustered in an interaction network centered on ENO1, PKLR, GAPDH, and TPI1, which are related to glycolysis. Thirteen GO functional annotations of MF, 97 of BP, and 23 functional annotations of CC were significantly enriched in the identified proteins. The principal KEGG pathways of the identified proteins were glycolysis/gluconeogenesis, carbon metabolism, biosynthesis of antibiotics, biosynthesis of amino acids, and metabolic pathways; therefore, these pathways played a key role in the effect of U251 cell-derived exosomes on hBMSCs. The identified proteins were involved in diverse biological processes and exhibited several molecular functions, mainly related to the activation of glycolysis/gluconeogenesis and metabolic pathways.

Energy metabolism involves energy production, release, conversion, and utilization. Normal cells generate energy mainly by aerobic oxidation of glucose [54]. In the presence of sufficient oxygen, tumor cells use glycolysis to generate energy. Although glycolysis is inefficient, it can provide ATP and macromolecules to meet the energy and material needs of the rapidly proliferating tumor cells [55]. The Warburg effect involves the conversion of energy production by tumor cells from oxidative phosphorylation to glycolysis, which is a major feature of cancer [56]. Tumor development and metastasis are closely related to glycolysis, and MSCs play an important role in the metabolic reprogramming of cancer cells and their stroma [57, 58]. Such abnormal metabolic reprogramming, particularly increased glycolysis, can induce the epithelial-mesenchymal transition in cancer cells and their acquisition of CSC-like properties, thereby promoting tumor progression [59].

Treatment with the U251 cell-derived exosomes resulted in the upregulation of Glut-1, HK-2, and PKM-2. This led to the increased glucose consumption and lactate and ATP generation, suggesting that U251 cell-derived exosomes enhanced the glucose metabolism of hBMSCs. Glut proteins transport glucose into cancer cells to supply the energy required for proliferation and differentiation via glycolysis or aerobic oxidation. Glut-1 is upregulated in a number of tumors and contributes to the Warburg effect [60]. HK-2 is the rate-limiting enzyme that catalyzes the first step of glycolysis, i.e., conversion of glucose into glucose-6-phosphate [61]. PK catalyzes the final step of glycolysis, the irreversible conversion of phosphoenolpyruvate into pyruvate, which is accompanied by ATP generation [62]. The PK isoform PKM-2 is commonly expressed in cancer cells and is involved in glycolysis, proliferation, and tumor-like phenotype transformation [63]. Treatment with the competitive inhibitor of glycolysis 2-DG reversed the effects of the U251 cell-derived exosomes on hBMSCs. In summary, inhibition of glycolysis may reverse the tumor-like phenotype transformation of hBMSCs in the glioma microenvironment.

## Conclusions

Our findings suggest that glioma cell-derived exosomes induce a tumor-like phenotype in hBMSCs, as indicated by the increased proliferation, migration, and invasion, and the expression of cancer markers. Proteomics and Western blot analyses showed that the exosome-induced tumor-like phenotype in hBMSCs was due to the activation of glycolysis. Therefore, glioma cell-derived exosomes promote the growth, migration, and invasion, as well as induce the tumor-like phenotype transformation, of hBMSCs by activating glycolysis (Fig. 13). Our findings suggest that exosomes activate MSCs in the tumor microenvironment, and the inhibition of this effect shows promise for the treatment of cancer.

**Fig. 13:** Exosomes derived from glioma U251 cells induce a tumor-like phenotype by promoting cell proliferation, invasion, and migration and expressing tumor-associated proteins, possibly through activating the glycolytic pathway in human bone marrow mesenchymal cells

## Abbreviations

1, 3-BPG: 1, 3-Bisphosphoglycerate
2-DE: Two-dimensional gel electrophoresis
2-DG: 2-Deoxy-d-glucose
AKT: Protein kinase B
ANXA2: Annexin A2
CAFs: Cancer-associated fibroblasts
CCK-8: Cell Counting Kit-8
CSCs: Cancer stem cells
DAVID: Database for Annotation, Visualization, and Integrated Discovery
DMEM: Dulbecco’s modified Eagles medium
ENO1: Alpha-enolase
FBS: Fetal bovine serum
GAPDH: Glyceraldehyde-3-phosphate dehydrogenase
GFAP: Glial fibrillary acidic protein
Glut-1: Glucose transporter type 1
hBMSCs: Human bone marrow mesenchymal stem cells
HK-2: Hexokinase-2
IEF: Isoelectric focusing
KEGG: Kyoto Encyclopedia of Genes and Genomes
MSCs: Mesenchymal stem cells
OD: Optical density
PAGE: Polyacrylamide gel electrophoresis
PBS: Phosphate-buffered saline
PCNA: Proliferating cell nuclear antigen
PEP: Phosphoenolpyruvate
PI: Propidium iodide
PI3K: Phosphatidylinositol 3-kinase
PKLR: Pyruvate kinase PKLR
PKM-2: Pyruvate Kinase M2
SDS: Sodium dodecyl sulfate
TAGLN: Transgelin
Tsg101: Tumor susceptibility gene 101 protein
